RETRACTED

# Acupuncture in the Treatment of Parkinson's Disease with Sleep Disorders and Dose Response

**DOI:** 10.1155/2022/7403627

**Published:** 2022-02-23

**Authors:** Lihong Li, Xiaoqing Jin, Wenjie Cong, Tingting Du, Wei Zhang

**Affiliations:** ^1^Department of Acupuncture, The Second Affiliated Hospital of Zhejiang Chinese Medical University, Hangzhou 310000, China; ^2^Department of Acupuncture, Zhejiang Hospital, Hangzhou 310007, China; ^3^Department of Acupuncture, The First Affiliated Hospital of Wenzhou Medical University, Wenzhou 325000, China; ^4^Department of Rehabilitation, Dongyang Traditional Chinese Medicine Hospital, Jinhua 322100, China; ^5^The Second Affiliated Hospital of Zhejiang Chinese Medical University, Rehabilitation & Sports Medicine Research Institute of Zhejiang Province, Hangzhou 310000, China

## Abstract

Acupuncture can effectively improve the sleep state, and most PD patients have sleep disorders. In this study, we used acupuncture to intervene in the sleep state of PDSD, so as to observe the changes and dose effect of Acutreatment on PDSD. 57 patients with PDSD, during medical treatment, aged 40–70 years were recruited to enroll in this trial. Each participant completed one condition, namely, Acutreatment (*n* = 30) and sham Acutreatment (placebo, stick flat needle on skin, *n* = 27). The Acutreatment was applied for 30 min once a day for a 30-day observation. UPDRSIII scores for motor symptom assessment and sleeping quality were assessed by PDSS-2, ESS as well as ActiGraph. Scale evaluation was made on the first day of admission and the thirtieth day. There were significant differences on all outcome indicators, except UPDRSIII, on day 30 compared with day 1 (*P* < 0.01). Compared with sham Acutreatment therapy, Acutreatment therapy has better performance in sleep latency, total sleep time, and sleep efficiency (*P* < 0.01). ActiGraph indicated that sleep efficiency of sham or Acutreatment in day 6 was significantly lower than that in day 5 (*P* < 0.05 and *P* < 0.01) and Acutreatment in day 7 was significantly lower than that in day 6 (*P* < 0.01). The sleep efficiency of Acutreatment in days 5, 6, and 7 was significantly higher than that in sham Acutreatment (*P* < 0.01). Moreover, Acutreatment in days 26, 27, and 28 was significantly higher than that in sham Acutreatment (*P* < 0.01). There was a close correlation between the difference of UPDRSIII and PDSS-2 (*r* = 0.5090, *P* < 0.05), sleep latency (*r* = 0.7201, *P* < 0.01), TST (*r* = −0.6136, *P* < 0.01), and sleep efficiency (*r* = −0.6707, *P* < 0.01). The sleep condition of PDSD patients can be improved by acupuncture, which can effectively relieve sleep quality, can also be shown by ActiGraph, and shows a dose-response relationship. Future research should explore Acutreatment with a larger sample size and compare the Acutreatment protocol goal formation of the system scheme.

RETRACTED

## 1. Introduction

Parkinson's disease (PD) is the most popular neurodegenerative disease up to date [1, 2]. Sleep disturbance is the chief complaint of 64.1% of PD patients [3]. There are various forms of Parkinson's disease sleep disorders (PDSD), such as annoying nighttime off symptoms, hallucinations, RBD (rapid eye movement sleep behavior disorder), RLS (restless legs syndrome), sleep apnea syndrome, or nocturia. Sleep disorders were positively correlated with PD motor disorders [4]. The main treatment of sleep disorders is oral medication [5]. Sleep medicines are widely used but may cause adverse reactions in patients with PD, such as nocturia, depression, hallucination, and dependence [6], or even aggravate sleep disorders through the use and toxicity of sleep drugs. Therefore, nondrug therapy has attracted more and more attention and is recommended as the first-line therapy before starting drug therapy. Acupuncture, as a common supplementary and placement therapy for PD, is used by 25.7%-76% of Parkinson's disease patients [7, 8]. Acupuncture treatment of sleep disorders has been affirmed in a great quantity of clinical studies [9, 10]. Nevertheless, recent trials of nondrug treatment trials for sleep disorders in PD patients are limited in quantity and poor in quality [11]. Therefore, it is urgent to explore the efficacy and dose effect of acupuncture in the treatment of PDSD.

We found in previous clinical observations that acupuncture is effective and has a dose effect in improving sleep. This study targets to comparatively investigate the treatment efficacy of Acutreatment on PDSD patients and to compare it with sham Acutreatment, to observe whether acupuncture is a placebo effect, whether acupuncture can indirectly improve motor symptoms while improving sleep quality of PDSD patients, and whether acupuncture has a dose-effect relationship.

## 2. Materials and Methods

### 2.1. Participants

This study was a single-center, randomized controlled (60 patients were randomly assigned according to a 1 : 1 ratio) clinical trial in PDSD wherein PD diagnosis was determined by their neurologist using UK brain bank criteria while taking levodopa or other Parkinson's drugs (equivalent dose of levodopa is greater than or equal to 300 mg/day). Individuals with PDSD met the Hoehn-Yahr 1.5-3.5, PSQI > 10, and the dose of sleep-regulating drugs was stable at least 28 days before consultation [12, 13]. Participants were excluded if they were diagnosed with cognitive impairment based on the Mini-Mental State Examination (MMSE) [14, 15], severe depression (Montgomery − Asberg Depression Scale > 34), alcohol or narcotic abuse, epilepsy history, participation in other clinical trials, and poor compliance: loss of more than 8 times in 26 treatments in the study.

RETRACTED

The trial was conducted in accordance with the guidelines of the Helsinki Declaration, approved by the Institutional Ethics Committee of the Zhejiang Provincial People Hospital (2019KY209) and registered on clinical trials (Registration No. ChiCTR1900022995). Each patient signed a written informed consent.

A total of 60 patients with PD, aged 40 to 70 years, were admitted in this study. The patients' gender, age, duration of disease (PD and SD/sleep disorders), UPDRSIII (“on” stage), Hoehn-Yahr staging, PSQI, and levodopa equivalent dose (LED) were evaluated. The sociodemographic and clinical characteristics of the participants are shown in Table 1.

### 2.2. Experimental Procedure

Sufferers were diagnosed by well-experienced evaluators who completed the Hoehn-Yahr staging, UPDRSIII, and PSQI scale. After the initial screening, participants were assigned to two conditions according to the random number table method: Acutreatment and sham Acutreatment (placebo). The Acu-group was treated for 30 min using acupuncture. In the sham Acu-group, participants maintain 30 min with a flat-headed needle placed in the same locations.

### 2.3. Treatment Protocol

*Acutreatment*: acupuncture needle (model: *Φ* 0.18 × 25 mm, Maanshan Bond Medical Instruments Co., Ltd., China); *points*: Shenting (GV24), Baihui (GV20), Zhaohai (KI6) and Guanyuan (GB20), 30 minutes each time, and the depth of needling is based on Deqi and applied during 30 min using once a day (except day 5, 6 and 28, 29 after admission), for a 30-day observation.

*Sham Acutreatment*: the needles, treatment method, points, and times are the same as above, but the flat-head needle needling is not percutaneous.

### 2.4. Efficacy Evaluation

*Motor symptom assessment*: UPDRSIII is the third part of the unified PD rating scale. It is used to assess the motor symptoms of Parkinson's disease. 14 items are used to evaluate the symptoms of Parkinson's disease including rotation movement, leg flexibility, gait, posture stability, low body movements, and standing. The scores were evaluated before enrollment and after the end of treatment in the “on period.”

*Sleeping quality evaluation*: Parkinson's disease Sleep Scale 2nd version (PDSS-2) is used for sleep quality and the Epworth Sleepiness Score (ESS) for “daytime sleepiness.”

PDSS-2 was developed and published in 2011 [16]. It consists of 15 projects evaluating three domains. Each domain composes of clusters of five questions (motor symptoms at night: 4, 5, 6, 12, and 13; PD symptoms at night: 7, 9-11, and 15; and disturbed sleep: 1-3, 8, and 14) [16]. Symptoms on each domain can be scored in the range of 0–20 points, whereas the sum of the 15 responses gives the total score of PDSS-2 with the maximum value of 60 points and higher scores meaning more nocturnal disturbance.

RETRACTED

ESS is a widely used measure of subjective daytime sleepiness. Dr. Johns first developed the ESS for adults in 1990 and subsequently modified it slightly in 1997. The ESS is a self-administered questionnaire with 8 questions. Respondents are asked to rate, on a 4-point scale (0-3), their usual chances of dozing off or falling asleep while engaged in eight different activities. The ESS score (the sum of 8 item scores, 0-3) can range from 0 to 24. The higher the ESS score, the higher that person's average sleep propensity in daily life (ASP) or their “daytime sleepiness,” The answer time of the questionnaire shall not exceed 3 minutes.

Sleep parameter detection was measured with ActiGraph (USA/wGT3X-BT, ActiGraph Corporation, Pensacola, FL, USA) for sleep latency, wake-up times, total sleep time (TST), sleep efficiency, which the patients wore on their nondominant wrist for 24 h/d throughout the course, and made three days before enrollment and days 5, 6, 7, 27, 28, and 29. Once returned, data were downloaded to a personal computer and manipulated in the ActiLife software version 6 (ActiGraph Corporation).

### 2.5. Statistical Analysis

Mean ± standard deviation ($\bar{x}\pm S$) was used to report sample characteristics and result measurement data. Descriptive statistics were used to calculate participant demographic and clinical characteristics. Several paired *t*-tests were completed in order to compare the outcome measures between conditions. SPSS 20.0 statistical software package was used for statistical analysis, *P* < 0.05.

## 3. Results

### 3.1. Participants

Of 87 patients who reported interest to take part in the trial, 60 individuals met the inclusion criteria and were assigned (Table 1). 3 participants withdrew in sham Acutreatment after the start of the intervention; thus, 57 individuals aged 40 to 70 years (33 women and 24men) were included. Baseline characteristics were similar between randomized groups at baseline, with the exception of the SF-36 sum score for mental health, where the control group had a higher (better) score (Table 1).

### 3.2. The Impact of Acutreatment on Motor and Sleeping Characteristics in PDSD Patients

We observed the UPDRSIII, PDSS-2, and ESS score on day 1 and day 30 of admission. We found that UPDRSIII had a trend of score loss in Acutreatment than that in sham Acutreatment on day 30 after the enrollment. However, there is no statistical significance (*P* > 0.05) (Figure 1(a)). Comparing the changes of PDSS-2 score on day 1, there was significant change on day 30 in the Acutreatment (*P* < 0.01), but there was no significant difference between Acutreatment and sham Acutreatment on day 30 (*P* < 0.05) (Figure 1(b)). The ESS score of Acutreatment was lower on day 30 than on day 1 (*P* < 0.01), and there was significant difference between Acutreatment and sham Acutreatment on day 30 (*P* < 0.01) (Figure 1(c)).

RETRACTED

Comparing the changes of sleep latency, TST, and sleep efficiency on day 1 and day 30, we found that there was significant change in sleep latency, sleep efficiency, and TST after treatment with Acutreatment (*P* > 0.01), and there was significant difference between Acutreatment and sham Acutreatment on day 30 (*P* < 0.01) (Figures 1(d)–1(f)).

### 3.3. Acutreatment Leads to Higher Sleep Efficiency with Dose-Effect Relationship

We observe the sleep efficiency change curve on the three days of admission (days -1, -2, and -3). We found that the sleep efficiency of sham or Acutreatment fluctuated between 60 and 70% (*P* > 0.05) (Figure 2(a)). But the sleep efficiency of sham or Acutreatment in day 6 was significantly lower than that in day 5 (*P* < 0.05 and *P* < 0.01), and Acutreatment in day 7 was significantly lower than that in day 6 (*P* < 0.01). The sleep efficiency of Acutreatment in days 5, 6, and 7 was significantly higher than that in sham Acutreatment (*P* < 0.01) (Figure 2(b)). From the figure, we can see that the sleep efficiency of Acutreatment in days 26, 27, and 28 was significantly higher than that in sham Acutreatment (*P* < 0.01) (Figure 2(c)).

### 3.4. Correlation between the Differences of UPDRSIII and PDSS-2, ESS, Sleep Latency, TST, and Sleep Efficiency in Acutreatment

There was a close correlation between the difference of UPDRSIII and PDSS-2 (*r* = 0.5090, *P* < 0.05), sleep latency (*r* = 0.7201, *P* < 0.01), TST (*r* = −0.6136, *P* < 0.01), and sleep efficiency (*r* = −0.6707, *P* < 0.01) in day 1 and day 30 (Figures 3(a)–3(e)).

### 3.5. Real-Time Effects of Acutreatment by ActiGraph

From the picture, we can see that PDSD had a bad sleep condition before treatment (days -3, -2, and -1). But PDSD has a good sleep condition on the 5th day (treatment day), and the sleep quality gets worse on days 6 and 7 (treatment cessation). Based on ActiGraph observation on days 26, 27, and 28 (treatment cessation on days 26 and 27), the sleep state in Acutreatment was close to normal (Figure 4).

RETRACTED

## 4. Discussion

The pathogeny of PDSD may be multifactorial, including degeneration of the central sleep regulatory area, the adverse effects of anti-Parkinson's drugs, age-related sleep changes, and the effects of dyskinesia (nocturnal motor disorders, motor disorders, tremors, and stiffness) [17]. In particular, motor symptoms and sleep disorders promote each other. On the one hand, the motor symptoms of PD can aggravate sleep disturbances. The neurochemical and structural changes of sleep awakening in PD can affect the regulation of sleep awakening. These changes are usually aggravated with the progress of disease [18]. The poor quality of sleep at night can promote the occurrence and development of dyskinesia in PD [4]. Therefore, improving the sleep quality of PD may help to relieve the motor symptoms of PD patients and improve life quality of PD. The types of PDSD include insomnia, sleep fragmentation, nocturnal urine, vivid dreams, circadian rhythm disorders, and excessive daytime sleepiness (EDS) [19]. Sleep drug use is not ideal for the improvement of sleep disorders, and it is easy to be addicted. Excessive daytime drowsiness (EDS) and nocturnal sleep disorder are common and debilitating symptoms of PD, but there is no effective treatment [20]. Long-term use will lead to drug resistance and may even produce or aggravate night dyskinesia in Parkinson's disease [21]. PD patients with sleep disorders not only affect the life treatment and motor symptoms of PD patients but also affect the life treatment of caregivers. Due to the uncertainty of etiology, the current symptomatic treatment cannot meet the clinical needs. As a kind of complementary therapy, acupuncture can increase the activity of the 5-HT nervous system [22], thus increasing sleep time and improving sleep quality.

A-B Classic of Acupuncture and Moxibustion points out that Yin-Yang Qiao meridians mainly manage limb activity, eyelid opening-closing, and sleep. Baihui and Shenting are acupoints of the Du meridian, which can calm the nerves. We use the acupoints of Shenmai, Zhaohai, Shenting, and Baihui to investigate the effects of acupuncture on the sleep condition of individuals with PDSD and the dose-effect correlation, which combines the functions of the Du meridian and the Qiao meridian and the circulation of meridians. Our findings suggest that compared with sham Acutreatment, Acutreatment can significantly improve sleep quality, such as the sleep efficiency, total sleep time, sleep latency, and daytime sleepiness in PDSD patients. In this study, sleep is positively correlated with improvement of motor symptoms, but the improvement of motor symptoms alone did not show statistical significance, which may be related to the small sample size and short study period. Acupuncture treatment of Parkinson's disease sleep disorder does show a dose-response relationship. It can show good results for the first time after acupuncture treatment, but after stopping treatment, it shows a gradual decline in efficacy until disappearance. However, when the maintenance treatment was continued to 25 days, it was found that stopping the treatment can still maintain the original effect, but as to how long this effect can be maintained, we need to observe in a further study.

RETRACTED

## 5. Conclusion

In this trial, Acutreatment can improve sleep condition in patients with PDSD in comparison to sham-Acu. Future trials should reveal the use of larger-sample cross-designed Acutreatments and compare deep-water Acu to identify the possibility of Acutreatment in improving the sleep status and delaying the development of motor symptoms in patients with PDSD. Follow-up of the dose-effect relationship presented by Acutreatment is required. Although the current research is still limited, the role of acupuncture in PDSD should not be underestimated. It has good safety and cost effectiveness.

## Figures and Tables

**Figure 1:** Impact of acupuncture on motor and sleeping characteristics in PDSD patients. Comparison of acupuncture-treated PD patients and sham-treated PD patients regarding motor symptoms ((a) UPDRSIII score) and sleeping parameters (b–f) on day 1 and day 30, respectively. The Acutreatment group is shown in blue, *n* = 30; the sham Acutreatment group is shown in red, *n* = 27. Statistics: comparison between groups: ^∗^*P* < 0.05 and ^∗∗^*P* < 0.01; comparison within groups: ^##^*P* < 0.01.

**Figure 2:** Acupuncture leads to increased sleep efficiency in a dose-dependent manner. Sleep efficiency rates were monitored by ActiGraph and are shown for the Acutreatment group (blue, *n* = 30) and the sham Acutreatment group (red, *n* = 27). (a) Before treatment start (days -3 to -1); (b) after start, during the first treatment intermission (days 5/6) plus the first of acupuncture reonset (day 7); (c) after start, during the second treatment intermission (days 26/27) plus the first of acupuncture reonset (day 28). Statistics: comparison between groups: ^∗^*P* < 0.05 and ^∗∗^*P* < 0.01; comparison within groups: ^##^*P* < 0.01.

**Figure 3:** Correlation of motor characteristic modifications and sleep quality improvement. Correlations of motor characteristic modifications and sleep quality parameter improvement are calculated as follows: data values were obtained by subtraction of sleep quality data values of day 30 from data values of day 1 (Figure 1). Motor characteristic (UPDRSIII score) data values were calculated analogously and are plotted against sleep quality parameter values in diagrams (a–e): (a) PDSS-2 (*r* = 0.5090, *P* < 0.05), (b) ESS (*r* = 0.1133, *P* > 0.05), (c) sleep latency (*r* = 0.7201, *P* < 0.01), (d) TST (*r* = −0.6136, *P* < 0.01), and (e) sleep efficiency (*r* = −0.6707, *P* < 0.01). Each data point represents a patient of the Acutreament group (*n* = 14–17, data points of patients with UPDRSIII subtraction values > 0 are not shown).

RETRACTED

**Figure 4:** Real-time effects of acupuncture on sleep efficiency. ActiGraph diagrams monitoring the sleep efficiency of a representative patient from the Acutreatment group on day -3 to day -1 before treatment start and after treatment start, on days when acupuncture was interrupted (days 5/6 and days 26/27), and the first day of treatment reonset (day 7 and day 28). Blue peaks represent activity; *x* − axes = time: 24 hours of ActiGraph measurement, with focus on the night time (vertical white dotted line = midnight).

**Table 1:** Comparison of baseline data between 2 groups.

Variables	Acutreatment (*n* = 30)	Sham Acutreatment (*n* = 27)
Gender (M/F)	13/17	11/16
Age (y, mean ± SD)	63 ± 6.73	59 ± 9.28
Duration of PD (y, mean ± SD)	5.94 ± 1.64	5.92 ± 1.68
Duration of SD (y, mean ± SD)	6.41 ± 2.83	5.92 ± 2.57
UPDRSIII (score, mean ± SD)	18.71 ± 2.14	19.58 ± 3.12
H-Y (stage, mean ± SD)	2.68 ± 0.39	2.67 ± 0.39
PSQI (score, mean ± SD)	14.71 ± 2.20	15.00 ± 2.13
LED (mg, mean ± SD)	352.91 ± 17.86	331.25 ± 38.91

## Data Availability

The data used to support the findings of this study are available from the corresponding author upon request.
